The article "Optimization of Machine Online Translation System Based on Deep Convolution Neural Network Algorithm" was retracted in 2023. Reasons: suspected computer-generated content; unreliable results or conclusions; concerns about the data; concerns about the results or conclusions.

# Optimization of Machine Online Translation System Based on Deep Convolution Neural Network Algorithm

**DOI:** 10.1155/2021/7388825

**Published:** 2021-09-29

**Authors:** Juan Zhao

**Affiliations:** School of Foreign Studies, North China University of Water Resources and Electric Power, Zhengzhou, Henan 450046, China

## Abstract

In order to effectively optimize the machine online translation system and improve its translation efficiency and translation quality, this study uses the deep separable convolution neural network algorithm to construct a machine online translation model and evaluates the quality on the basis of pseudo data learning. In order to verify the performance of the model, the regression performance experiment of the model, the method performance experiment of generating pseudo data for specific tasks, the sorting task performance experiment of the model, and the machine translation quality comparison experiment are designed. RMSE and MAE were used to evaluate the regression task performance of the model. Spearman rank correlation coefficient and delta AVG value were used to evaluate the sorting task performance of the model. The experimental results show that the MAE and RMSE values of the model are decreased by 2.28% and 1.39%, respectively, compared with the baseline system under the same experimental conditions, and the Spearman and delta AVG values are increased by 132% and 100.7%, respectively, compared with the baseline system. The method of generating pseudo data for specific tasks needs less data and can make the translation system reach a better level faster. When the number of instances is more than 10, the quality score of the model output is higher than that of Google translation whose similarity is more than 0.8.

## 1. Introduction

Machine online translation system is to translate a source language into another target language by combining artificial intelligence technology and human language processing technology. The machine online translation system can realize the translation of multiple languages, its efficiency is far higher than that of manual translation, and it is easier to use. In the context of globalization, the Machine online translation system plays a positive role in promoting economic exchanges and mutual understanding among people all over the world [1]. In most cases, the quality of machine translation is lower than that of manual translation. In the professional field, the accuracy of machine translation is still low [2]. How to improve the accuracy of the machine translation system through deep learning is one of the important research directions. In addition, language translation and image translation are also in the research stage. The main content of this study is to establish an Machine online translation model based on the deep separable convolutional neural network algorithm, provide deep learning and training methods, improve the quality of translation system model and translation, and reduce the dependence of the translation system on manual annotation.

The article "Optimization of Machine Online Translation System Based on Deep Convolution Neural Network Algorithm" was retracted in 2023. Reasons: suspected computer-generated content; unreliable results or conclusions; concerns about the data; concerns about the results or conclusions.

Some achievements have been made in the research of the online translation model. At present, the main technologies of online translation model are neural network algorithm, cloud computing model, PDCA translation method, and so on. Chen designed a new machine-aided translation system [3]. The system hardware is divided into four layers: user layer, business layer, computing layer, and storage layer. The storage structure, translation structure, and retrieval structure are designed, respectively. The results show that the machine-aided translation system based on cloud computing costs less time than the traditional translation system. Gao and Liu proposed PDCA translation method which is the PDCA cycle translation mode of P (plan), D (do), C (check), and a (action). In the process of translation, UGC online translation is subject to pretranslation quality evaluation, preediting, term management, and positioning so as to fundamentally ensure the translation quality, and a translation quality management flow chart for user generated content is proposed, which plays a significant role in promoting the orderly development of circular translation mode translation [4]. The specific operation mode is to start from the translation of UGC (user generated content) sample text and carry out quality evaluation, preediting, term management, and positioning of UGC online translation in the process of translation so as to ensure the quality of translation and put forward the flow chart of translation quality management for user generated content. The neural network algorithm translation system is mainly based on deep learning, which is a branch of machine learning. Compared with traditional machine learning methods, deep convolution neural network has a deeper network structure, and its operation efficiency and accuracy have significant advantages. These deep structures closely imitate the biological process of vision. Through the establishment of a system with visual features and a series of “convolution” operations to complete the deep learning, the results show that the extracted features can well represent the quality of the image [5]. The online translation model needs model performance evaluation and translation quality evaluation, and attention should be paid to noise interference in the process of experiment [6].

The article "Optimization of Machine Online Translation System Based on Deep Convolution Neural Network Algorithm" was retracted in 2023. Reasons: suspected computer-generated content; unreliable results or conclusions; concerns about the data; concerns about the results or conclusions.

There are two innovations in this study. The first is the optimization of the algorithm. The use of the deep separable convolution neural network algorithm can improve the efficiency of convolution operation. The second is the specific task pseudo data acquisition mode based on deep learning, which can reduce the amount of manual annotation and improve the training efficiency. The second part is the establishment and optimization of the online translation system model. The third part is the main model test design, including parameter setting, performance evaluation method, and standard setting. The fourth part is the analysis of the experimental results.

## 2. Establishment and Optimization of Machine online translation Model Based on Deep Convolution Neural Network Algorithm

This paper uses the deep convolution network algorithm shown in the title to establish the model, translate the original language, and output the target language. Because the output result is language, the language cannot be compared intuitively, so the model needs to be further improved.

### 2.1. The Establishment of Online Translation Model of Neural Network Algorithm

The neural network translation model can be directly mapped to the output sequence in an end-to-end way [7]. The translation structure of the neural network algorithm model is shown in Figure 1.

The model consists of two parts: an electronic encoder and a decoder. Suppose the source language of the given point is as follows:

(1) $$\begin{array}{c} X=\left\{x_{1},x_{2},\ldots ,x_{n}\right\}. \end{array}$$

The target language settings are shown in the following formula:

(2) $$\begin{array}{c} Y=\left\{y_{1},y_{2},\ldots ,y_{n}\right\}. \end{array}$$

Then, the model translation probability based on neural network can be expressed as follows:

(3) $$\begin{array}{c} p\left(Y|X\right)=\prod_{t=1}^{m}P\left(yt|y<t,X\right). \end{array}$$

In formula (3), *t*=*y*_1_, *y*_2_,…, *y*_*t*−1_, and GRE and other nonlinear elements are integrated into the deep convolution neural network model to obtain the hidden state *h*_*t*_ as follows:

(4) $$\begin{array}{c} h_{t}=\text{RNN}\left(h_{t-1},x_{t}\right). \end{array}$$

According to the context information, the final hidden state is obtained by integrating the coding results of different directions. The calculation of this process is shown in the following formulas:

(5) $$\begin{array}{c} {\overset{⟶}{h}}_{t}=\text{RNN}\left({\overset{⟶}{h}}_{t-1},x_{t}\right), \end{array}$$

(6) $$\begin{array}{c} {\overset{\leftarrow }{h}}_{t}=\text{RNN}\left({\overset{\leftarrow }{h}}_{t-1},x_{t}\right), \end{array}$$

(7) $$\begin{array}{c} h_{t}=\left[\frac{{\overset{⟶}{h}}_{t}}{{\overset{\leftarrow }{h}}_{t}}\right]. \end{array}$$

The hidden state is finished by the final decoder end. The algorithm is shown in the following formulas:

(8) $$\begin{array}{c} q=g\left(y_{t-1},c_{t},s_{t}\right), \end{array}$$

(9) $$\begin{array}{c} p\left(y_{t}|y<t,X\right)=\text{softmax}\left(q\right). \end{array}$$

In formula (8), *q* is the word tensor of the target end to be measured; *g*(·) represents a nonlinear element; *s*_*t*_ is the hidden state of the decoder; *c*_*t*_ represents the weighted sum of source hidden states as given in the following formula:

(10) $$\begin{array}{c} c_{t}=\text{attention}\left(s_{t-1},h\right)=\sum_{i=1}^{n}a_{t,i}h_{i}, \end{array}$$

(11) $$\begin{array}{c} a_{t,i}=\text{softmax}\left(V_{a}^{T}\tanh\left(W_{a}s_{t-1}+U_{a}h_{j}\right)\right). \end{array}$$

In the formula, *V*_*a*_, *W*_*a*_, and *U*_*a*_ are all training parameters of the neural network model.

The article "Optimization of Machine Online Translation System Based on Deep Convolution Neural Network Algorithm" was retracted in 2023. Reasons: suspected computer-generated content; unreliable results or conclusions; concerns about the data; concerns about the results or conclusions.

### 2.2. Online Translation Model for Optimization of Deep Convolutional Neural Network Algorithm

The online translation model based on the neural network algorithm is optimized, and a new deep separable convolutional neural network algorithm is adopted [8]. The depth separable convolution neural network algorithm divides the traditional convolution into depth convolution and point by point convolution. Its structure is shown in Figure 2.

As shown in Figure 2, in the deep convolution layer, each input channel performs spatial convolution independently, each convolution core is responsible for its own channel, and each channel performs convolution operation corresponding to a specific convolution core. This deep convolution algorithm learns each channel separately, instead of corresponding to the same filter, so it can extract better features. Point by point convolution uses a 1 *∗* 1 convolution window to expand the convolution operation and maps the output of deep convolution to a new channel space [9]. In traditional convolution layer, feature extraction and feature fusion are carried out at the same time, which requires many parameters and low efficiency. The depth volume integration is divided into two steps: depth convolution and point-to-point convolution; that is, feature extraction and feature fusion are carried out step by step. The use of model parameters is less, the parameters can be more fully used for learning, and the operation efficiency can be further improved. The deep convolution neural network algorithm can maximize the use of parameters to complete network training and feature extraction in the case of few parameters. Compared with other neural network algorithms, its accuracy and efficiency are higher. The NMT model based on the deep separable convolutional neural network algorithm proposed in this study is based on the NMT model of attention mechanism, and the deep separable convolutional neural network is integrated into the input layer and coding layer [10]. After the convolution operation in the input layer, the data enter the encoder for encoding operation. The structure of the encoder is shown in Figure 3.

The article "Optimization of Machine Online Translation System Based on Deep Convolution Neural Network Algorithm" was retracted in 2023. Reasons: suspected computer-generated content; unreliable results or conclusions; concerns about the data; concerns about the results or conclusions.

As shown in Figure 3, the encoder is composed of NX identical layers; each layer can be divided into two sublayers: the first sublayer is self attention layer and the second sublayer is feedforward neural network layer. The output results of the first sublayer and the second sub layer are, respectively, sent to two different summation and normalization layers for separate processing [11]. The summation and normalization layer consists of two steps. The first step is residual connection, and the second step is layer standardization. The decoder architecture of summation and normalization layer is basically the same.

### 2.3. Translation Quality Estimation Method

The translation output of machine online translation needs to be evaluated by the quality evaluation model [12, 13]. Based on the classical recurrent neural networks (NNs), a memory cell structure is proposed. Each memory unit is divided into four parts: an input gate, an output gate, a forgetting gate, and a self cyclic connection.

The translation quality estimation model uses the vector representation of the source language sentence and the vector representation of the translation to estimate the quality of the translation. The structure of the translation quality estimation model is shown in Figure 4.

As shown in Figure 4, it is the structure of the translation quality estimation model, and its algorithm content is as follows: the two sentence vectors obtained by bidirectional recurrent neural network are expressed as *ctx*_*x*_ and *ctx*_*y*_, and these two expressions are used to generate new vectors, respectively, *V*_*x*_, *V*_*y*_ as follows [14, 15]:

(12) $$\begin{array}{c} V_{x}=\sigma \left(W_{x}*ctx_{x}\right), \end{array}$$

(13) $$\begin{array}{c} V_{y}=\sigma \left(W_{y}*ctx_{y}\right). \end{array}$$

In formulas (12) and (13), *W*_*x*_ and *W*_*y*_ represent the weight of two sentence vectors *V*_*x*_ and *V*_*y*_, respectively, and score(*X*, *Y*)=1 − cos(*V*_*X*_, *V*_*Y*_) and cos(*V*_*X*_, *V*_*Y*_)=(*V*_*X*_ · *V*_*Y*_/‖*V*_*X*_‖*∗*‖*V*_*Y*_‖).

The cosine distance between sentence vectors *V*_*x*_ and *V*_*y*_, as a predictor of translation quality, is expressed in the following formulas:

(14) $$\begin{array}{c} \text{score}\left(X,Y\right)=1-\cos\left(V_{X},V_{Y}\right), \end{array}$$

(15) $$\begin{array}{c} \cos\left(V_{X},V_{Y}\right)=\frac{V_{X}\cdot V_{Y}}{\left\|V_{X}\right\|*\left\|V_{Y}\right\|}. \end{array}$$

In formula (14), score is the 2-norm of the sentence vector DeltaAvg_*v*_=(∑_*n*=2_^*N*^DeltaAvg_*v*_[*n*]/*N* − 1) and *S*_*i*,*j*_=∪_*k*=1_^*j*^*S*_*k*_ is the 2-norm of the sentence vector *V*(*S*).

The article "Optimization of Machine Online Translation System Based on Deep Convolution Neural Network Algorithm" was retracted in 2023. Reasons: suspected computer-generated content; unreliable results or conclusions; concerns about the data; concerns about the results or conclusions.

### 2.4. Model Training Method

The translation quality estimation model needs training and deep learning; in the process of training, it needs a lot of manual annotation data. In the process of Machine online translation, there are not many opportunities to obtain annotated data, and the effect of training the model in a small training set is not ideal. In view of this situation, this study proposes a data generation method of the bilingual parallel corpus method, which can use parallel expected random production data to pretrain the online translation model. Then, the real training set is used to adjust or fine tune the parameters of the online translation model [16]. In the pretraining process, the dynamic learning rate gradient random descent method is used to update the model parameters, and the updated parameters will be used as the initialization parameters in the adjustment or fine-tuning stage. In order to ensure the effectiveness of training data generation, this study uses the pseudo data generation model training algorithm in the training. The algorithm can generate the corresponding pseudo data for a specific task, avoiding the defects of low accuracy and pertinence of training data caused by the random generation of pseudo data. The detailed process of generating targeted pseudo data is shown in Figure 5.

As shown in Figure 6, the generation process of targeted pseudo data can be divided into the following three steps. (1) The error translation of development set is analyzed, and the errors in translation include four text editing errors, including insertion error, deletion error, replacement error, and reordering error. By analyzing the number and score of these four kinds of errors, we can get the error translation distribution characteristics of the development set [17]. (2) Similar sentence retrieval: each sentence in the development set can be searched from a large-scale bilingual parallel corpus, and *N* sentences most similar to the sentences in the development set can be found. These *n* sentences form a set, which is called candidate bilingual sentence pair set [18]. (3) Pseudo translation generation and scoring: for candidate bilingual sentences, *n* sentences in the set are edited according to the error distribution characteristics of the development set to generate pseudo translation. The quality score of the pseudo translation is generated by comparing the pseudo translation with the standard translation. The calculation of four text editing errors required for scoring is shown in Table 1.

The article "Optimization of Machine Online Translation System Based on Deep Convolution Neural Network Algorithm" was retracted in 2023. Reasons: suspected computer-generated content; unreliable results or conclusions; concerns about the data; concerns about the results or conclusions.

## 3. Experimental Method of Deep Convolution Neural Network Algorithm for Machine Online Translation Model

### 3.1. Experimental Conditions and Parameter Setting of Deep Convolution Neural Network Algorithm for Machine Online Translation Model

This experiment uses the English Chinese sentence level quality estimation task data published by WMT2015 to compare the deep convolution neural network algorithm translation model established in this study with the baseline system. The experimental parameters are shown in Table 2.

As can be seen from Table 2, the pretraining data of the deep convolution neural network algorithm for the machine online translation model contain about 1970k English Chinese data, and the fine-tuning training contains 12711 source language sentences. These source language sentences come from the sentence level quality estimation task in the training set, and each source language information has its corresponding machine translation translation and corresponding manual postediting translation. There are 1718 sentences in the test set. The source language sentences come from the test set sentences of the sentence level quality estimation task. Every day, the source language sentences have their corresponding machine translation translations and corresponding manual postediting translations. HTER score was used to evaluate the translation, and the score was calculated by using the terp tool [19]. In addition, in the process of model training, the parameters of the word representation vector are not adjusted. The hidden layer unit of the bidirectional recurrent neural network is 1000, the context vector unit is 200, and the word representation dimensions of the source language and the target language are set to 512. The size of each batch is set to 100 in the pretraining process and 50 in the fine-tuning process [20].

### 3.2. Experimental Evaluation Method of Deep Convolution Neural Network Algorithm for Machine Online Translation Model Performance

In this study, four evaluation criteria are mainly used. The mean absolute error (MAE) represents the mean absolute error between two sample groups [21]. Root mean square error (RMSE) is used to calculate the root mean square error between two sample groups. The larger the coefficient is, the better the correlation is. Delta AVG can be expressed in the following formulas:

(16) $$\begin{array}{c} {\text{DeltaAvg}}_{v}\left[n\right]=\frac{\sum_{k=1}^{n-1}V\left(S_{1,k}\right)}{n-1}-V\left(S\right), \end{array}$$

(17) $$\begin{array}{c} {\text{DeltaAvg}}_{v}=\frac{\sum_{n=2}^{N}{\text{DeltaAvg}}_{v}\left[n\right]}{N-1}, \end{array}$$

*S*_*i*,*j*_=∪_*k*=1_^*j*^*S*_*k*_ is defined in formula (16). *V*(*S*) represents the quality score of sentence *s*, and *V*(*S*)(*s* ∈ *S*) represents the average of the quality score of all sentences *s*. The larger the value of DeltaAvg_*v*_, the better the performance of the deep convolution neural network algorithm for the machine online translation model, and vice versa [22]. Among the four evaluation criteria, RMSE and MAE are used to evaluate the performance of regression task. The smaller the RMSE and MAE, the better the performance. Spearman rank correlation coefficient and delta AVG value are used to evaluate the sorting task performance of the model. The larger the value is, the better the performance is [23].

The article "Optimization of Machine Online Translation System Based on Deep Convolution Neural Network Algorithm" was retracted in 2023. Reasons: suspected computer-generated content; unreliable results or conclusions; concerns about the data; concerns about the results or conclusions.

Baseline comparison method and BLEU method were used in the evaluation. The baseline comparison method is to translate the source language sentences in the baseline system by the machine translation model and then compare the machine translation with the baseline system translation. In the baseline system, RBF kernel function is used to fuse multiple black box features. The black box features include the length of source language sentence, the length of target language sentence, the length of source language sentence, the number of target words appearing, the weighted average number of translations corresponding to the speech model, the weight of source language words, the probability of the source language sentence model, the probability of the target language sentence model, the number of punctuation in source language, the number of target words, and the number of punctuation in the target language. The theoretical basis of the BLEU method is that when there is a high similarity between the machine translation system and the manual translation, the quality of the machine translation can be considered as relatively high, and the higher the similarity, the higher the translation quality [24]. The specific evaluation method is to count the number of *n*-ary words in both machine translation and manual translation and calculate the number of these *n*-ary words and the total word data of machine translation. The value obtained is the evaluation result. The evaluation method is convenient and fast, but the accuracy is relatively low.

## 4. Experimental Results of Machine Online Translation Model Based on Deep Convolution Neural Network Algorithm

### 4.1. Performance Evaluation of Deep Convolution Neural Network Algorithm for Machine Online Translation Model Training Methods

This experiment compares the performance of different models in two aspects: regression task and sorting task. The experimental conditions of different models are the same. The RMSE and MAE performance values of regression task are obtained from the training results of regression task. See Table 3 for details. The smaller the RMSE and MAE values, the higher the regression degree and the better the performance of the model.

The article "Optimization of Machine Online Translation System Based on Deep Convolution Neural Network Algorithm" was retracted in 2023. Reasons: suspected computer-generated content; unreliable results or conclusions; concerns about the data; concerns about the results or conclusions.

From Table 3, the MAE and RMSE values of the experimental results of the deep convolution neural network algorithm for the machine online translation model can be seen.

The error of the system established in this study is greater than that of the baseline system, when the training set is used for training, which shows that the baseline system has certain advantages. When using direct training, the MAE and RMSE values of the experimental results are slightly less than the baseline system, while using training + fine-tuning mode, the MAE and RMSE values of the experimental results are significantly less than the baseline system, and the MAE and RMSE values of the baseline system are decreased by 2.28% and 1.39%, respectively. Spearman rank correlation coefficient and delta AVG will be obtained from the performance evaluation experiment of the model. The results are shown in Tables 4 and 5. The larger the Spearman rank correlation coefficient and delta AVG, the better the performance.

It can be seen from Table 4 that under the pretraining conditions of 50K, 100K, 200K, 500K, 1000K, and 1500K, the quality of pseudo data generated for specific tasks is better than that generated randomly. When the data size is 500K, the performance of the deep convolution neural network algorithm for the machine online translation model is the best, and the Spearman rank correlation coefficient is 0.319. When the performance of the model reaches a better level (Spearman rank correlation coefficient is not less than 0.245), the scale of training data needed for the way of generating pseudo data for specific tasks is small. When the scale of pseudo data generated for a specific task exceeds a certain value, the performance will decline, and the inflection point of the decline will be around 500K. It is speculated that the reason may be that there is a certain interference relationship between the pseudo data generated for a specific task, which is mutual noise. If the interference accumulates to a certain extent, the overall performance will decline. On the whole, the method of generating pseudo data for specific tasks, when selecting the appropriate data size for training, can more quickly make the model performance to a better level, and the overall level of the model has been improved.

The article "Optimization of Machine Online Translation System Based on Deep Convolution Neural Network Algorithm" was retracted in 2023. Reasons: suspected computer-generated content; unreliable results or conclusions; concerns about the data; concerns about the results or conclusions.

It can be seen from Table 5 that the Spearman and delta AVG values of the experimental results of the deep convolution neural network algorithm for the machine online translation model established in this study are less than those of the baseline system when the training set is used for pretraining, which shows that the baseline system has certain advantages. When using direct training, the Spearman and delta AVG values of the experimental results are significantly higher than those of the baseline system. When using pretraining and fine-tuning mode, the experimental results show that the values of Spearman and delta AVG are much higher than the baseline system, and the values of Spearman and delta AVG are increased by 132% and 100.7%, respectively, compared with the baseline system.

### 4.2. Comparison of the Quality of Deep Convolution Neural Network Algorithm for Machine Online Translation Model Output Translation

BLEU score was used to compare the translation quality of the model. In order to avoid large errors caused by too few examples and too much noise caused by too many examples, 150 examples were selected in this experiment to fuse the translations, which increased from 0 to 60. The ideal fusion upper limit of BLEU and the real BLEU score in each fusion case were calculated, respectively. In addition, the translation results of the model established in this paper are compared. When the similarity is greater than 0.8, the instance is replaced. The specific experimental results are shown in Figure 6.

It can be seen from Figure 6 that the upper limit of BLEU score increases with the increase in the number of instances, but the increase rate slows down with the further increase in instances. When the number of instances is small, the real BLEU value changes quickly. When the number of instances is more than 10, the machine translation score of the deep convolution neural network algorithm of the machine online translation model established in this paper is relatively high. With the further increase in the number of instances, the BLEU score of the consistency optimization model fluctuates slightly. It is speculated that with the increase in the maximum number of fusion instances, the number of translation instances of each sentence will fluctuate greatly. Therefore, in the process of machine translation, we should set a reasonable number of instances to avoid large fluctuations in the number of translation instances, resulting in large changes in system performance. The results of this study show that when the number of instances is about 10, a high-quality translation can be obtained, and the performance of the translation system is relatively stable. In order to further explore the translation performance of this algorithm and Google translation, this topic applies the two and the benchmark model to the translation comparison under different sentence lengths. The results are shown in Figure 7.

The article "Optimization of Machine Online Translation System Based on Deep Convolution Neural Network Algorithm" was retracted in 2023. Reasons: suspected computer-generated content; unreliable results or conclusions; concerns about the data; concerns about the results or conclusions.

According to Figure 7, when the sentence length is 0–10, the BLEU scores of the three models are high, and the accuracy of the algorithm in this paper is higher than that of Google translation, and the BLEU score of the benchmark model is the lowest. With the continuous decline in sentence length, the BLEU scores of the three models show a downward trend as a whole. This shows that the longer the length of the sentence, the more complex the dependency and the higher the difficulty of translation. Nevertheless, the algorithm in this paper still maintains superior translation performance, and its BLEU score decreases as a whole. However, in the process of continuous growth of sentence length, the BLEU score of the algorithm in this paper shows a certain recovery and is always higher than that of Google translation and benchmark model.

## 5. Conclusion

In this study, the machine translation system based on the neural network algorithm is improved, and the depth separable convolution neural network algorithm is used to establish the machine online translation model. In order to evaluate the quality of machine translation model output, a quality evaluation method based on pseudo data learning is adopted to reduce the amount of manual annotation data. For the generation of pseudo data in model training, this study proposes a pretraining + fine-tuning mode. In order to improve the quality of pseudo data generation, the method of generating pseudo data for specific tasks is adopted. In order to verify the performance of the model established in this study and the quality of the output translation, four groups of experiments are designed, which are as follows: the regression performance experiment of this system, the method performance experiment of generating pseudo data for specific tasks, the sorting task performance experiment of this system, and the quality comparison experiment of machine translation. The experimental results show that the MAE and RMSE values of the machine translation system model established in this study are decreased by 2.28% and 1.39%, respectively, compared with the baseline system under the same experimental conditions, and the regression performance is better than that of the baseline system; compared with the baseline system, Spearman value and delta AVG value are improved by 132% and 100.7%, respectively, and the performance is far better than baseline system. The method of generating pseudo data for specific tasks can make the translation system reach a better level faster with less data than the method of generating pseudo data randomly. The results of translation quality experiments show that when the number of instances is more than 10, the machine translation score of the model established in this study is higher than that of Google translation whose similarity is greater than 0.8.

The article "Optimization of Machine Online Translation System Based on Deep Convolution Neural Network Algorithm" was retracted in 2023. Reasons: suspected computer-generated content; unreliable results or conclusions; concerns about the data; concerns about the results or conclusions.

## Figures and Tables

**Figure 1:** Structure diagram of machine translation based on deep convolution neural network.

**Figure 2:** Deep separable convolutional neural network.

**Figure 3:** NMT encoder based on depth separable convolution.

**Figure 4:** Block diagram of the translation quality estimation model.

**Figure 5:** Generation process of targeted pseudo data.

**Figure 6:** The influence of the number of translation examples on the translation.

**Figure 7:** Comparison results of sentence translation performance under different lengths.

**Table 1:** Setting of task-specific generating pseudo data.

Operation	Number	Type	Position
Insert	Ratio of sentence length *∗* words to sentence length	Words not appearing in random selection sentences	Random
Delete	Ratio of sentence length *∗* words to sentence length	Words not appearing in random selection sentences	Random
Replace	Ratio of sentence length *∗* words to sentence length	Words not appearing in random selection sentences	Random
Sequence adjustment	Ratio of sentence length *∗* words to sentence length	Random generation of sequence length	Random

**Table 2:** Description of experimental parameters on the deep convolution neural network algorithm for the machine online translation model.

Data	Scale (sentence)	Describe
Pretraining	1970623	Source language, standard translation
Fine tuning	12711	Source language, machine translation translation, manual postediting of translation, HTER score
Test	1718	Source language, machine translation translation, manual postediting of translation, HTER score

**Table 3:** Performance comparison on regression task.

System	MAE	MAE decrease percentage%	RMSE	RMSE decrease percentage%
Baseline system	14.81	—	19.14	—
Deep convolution neural network algorithm for the machine online translation model	14.75	0.49	19.02	0.59
Direct training				
Deep convolution neural network algorithm for the machine online translation model	17.27	—	23.48	—
Pretraining				
Deep convolution neural network algorithm for the machine online translation model	14.49	2.28	18.87	1.39
Pretraining + fine tuning				

**Table 4:** Spearman-coefficients of training models with different pseudo data generation methods on the deep convolution neural network algorithm for the machine online translation model.

Data size (number of sentences) (K)	Machine translation	Randomly generated pseudo data	Generating pseudo data for specific tasks
50	0.138	—	0.188
100	0.149	—	0.247
200	0.248	0.248	0.248
500	—	0.248	0.319
1000	—	0.257	0.286
1500	—	0.259	0.282

The article "Optimization of Machine Online Translation System Based on Deep Convolution Neural Network Algorithm" was retracted in 2023. Reasons: suspected computer-generated content; unreliable results or conclusions; concerns about the data; concerns about the results or conclusions.

**Table 5:** Performance comparison of sorting tasks.

System	DeltaAvg	DeltaAvg decrease percentage%	Spearman	Spearman decrease percentage%
Baseline system	2.15	—	0.14	—
Deep convolution neural network algorithm for the machine online translation model	4.09	89.7	0.24	76.8
Direct training				
Deep convolution neural network algorithm for the machine online translation model	2.07	—	0.11	—
Pretraining				
Deep convolution neural network algorithm for the machine online translation model	5.03	132	0.28	100.7
Pretraining + fine tuning				

## Data Availability

The data used to support the findings of this study are available from the corresponding author upon request.
